This article has been retracted.

# Influence of the use of various imaging units and projections on the radiation dose received by children during chest digital radiography

**DOI:** 10.1371/journal.pone.0255749

**Published:** 2021-08-05

**Authors:** Hongrong Xu, Kaiping Huang, Bo Liu, Jinhua Cai, Huan Zheng, Helin Zheng, Qiurui Yang, Changhong Yao

**Affiliations:** 1 Department of Radiology, Children’s Hospital of Chongqing Medical University, Chongqing, China; 2 Ministry of Education Key Laboratory of Child Development and Disorders, Chongqing, China; 3 National Clinical Research Center for Child Health and Disorders, Chongqing, China; 4 Chongqing Key Laboratory of Pediatrics, Chongqing, China; Ministry of Natural Resources North Sea Bureau, CHINA

## Abstract

**Objective:**

To investigate the impact of the use of different imaging units and projections on radiation dose and image quality during chest digital radiography (DR) in 3- and 4-year-old children.

**Methods:**

Two hundred forty 3- and 4-year-old participants requiring chest DR were included; they were divided into three groups: supine anterior-posterior projection (APP), standing APP and standing posterior-anterior projection (PAP). Each group included 40 participants who were evaluated using the same imaging unit. The dose area product (DAP) and the entrance surface dose (ESD) were recorded after each exposure. The visual grading analysis score (VGAS) was used to evaluate image quality, and the longitudinal distance (LD) from the apex of the right lung to the apex of the right diaphragm was used to evaluate the inspiration extent.

**Results:**

DAP and ESD were significantly lower in the standing PAP and APP groups than in the supine APP group (*P*<0.05), but LD was significantly higher in the standing PAP and APP groups than in the supine APP group (*P*<0.05). Additionally, the pulmonary field area was significantly higher for the standing PAP group than for the standing and supine APP groups (*P*<0.05). The correlations between ESD, DAP, and VGAS were positive (*P*<0.001), showing that larger ESD and DAP correspond to higher VGAS. The correlations between ESD, DAP, and body mass index (BMI) were also positive (*P*<0.05), indicating that higher BMI corresponds to larger ESD and DAP. Finally, no differences in DAP, ESD, VGAS, LD, pulmonary field area, or BMI were noted between males and females (*P*>0.05).

**Conclusion:**

The radiation dose to superficial organs may be lower with standing PAP than with standing APP during chest DR. Standing PAP should be selected for chest DR in 3- and 4-year-old children, as it may decrease the required radiation dose.

## Introduction

Digital radiography (DR) is widely applied in diverse medical environments and plays an important role in reaching a definite diagnosis [1]. The thyroid, skin, and breast tissues of children are more radiosensitive than those of adults, and the possibility of radiation-induced cancer in children is approximately 2–3 times greater than that in adults [1–4]. In addition, 3- and 4-year-old children are susceptible to numerous respiratory tract diseases because of their physiological characteristics and because their immune systems are still developing. Chest DR is used in the radiologic diagnosis of respiratory illness in this population and can meet clinical needs [5]. Nonetheless, children are inclined to be uncooperative during chest DR, and the choice of a comfortable position for DR can therefore help guarantee a successful inspection and adequate image quality [4]. Supine anterior-posterior projection (APP) is often used with uncooperative children because it constrains their motion and reduces the risk of noneffective X-rays resulting from body motion during exposure. Standing APP is generally used with cooperative children because it allows observation of their breathing and relieves their angst. The standing posterior-anterior projection (PAP) is applied to very cooperative children and permits sufficient visualization of the pulmonary field [6]. Previous studies [7–10] principally employed various combinations of tube voltage and current (milliampere seconds, mAs) to optimize exposure parameters for chest DR. The dose area product (DAP) and the entrance surface dose (ESD) were used to evaluate the radiation dose received, and the visual grading analysis score (VGAS) was applied to evaluate image quality [4,5,7,9,10]. However, these methods have some restrictions. The primary restriction is that the age group is comparatively large (e.g., 1–3 years, 3–7 years) [8], and children in the same age group may have tremendous diversity in weight. Conversely, body size may vary substantially even among children with the same body weight [11–13]. Furthermore, some academicians have found an impact of body mass index (BMI) on the radiation dose received by adults undergoing thorax X-ray examination and a marked augmentation in the radiation dose for male patients compared to female patients [14]. However, few studies have specifically addressed whether sex, BMI, or the imaging unit and type of projection used in children influence the radiation dose and image quality. Hence, some academicians [4] have suggested using children’s age, height, and weight to obtain normative body sizes for some age ranges and applying these criteria to regulate exposure parameters and increase image quality.

In this study, we selected children within a small age range (3–4 years) as study subjects. Fixed, optimized exposure parameters and radiologic techniques were used based on the literature. We analyzed the impact of sex, type of imaging unit used, BMI, and type of photography projection on the radiation dose and image quality of chest DR in children.

## Materials and methods

### Ethics statement

The prospective study protocol was approved by the ethics committee of the Children’s Hospital of Chongqing Medical University. Written informed consent was obtained from the parents or other legal guardians of each participant before the examinations. All parents or guardians of the participants provided written informed consent in accordance with the Declaration of Helsinki.

### Participants

A total of 488 participants who were referred for chest DR at our institution from July to December 2019 were enrolled in this study. Due to the prospective study protocol using isodistance sampling, the participants who exhibited good cooperation were divided into a supine APP group, a standing APP group and a standing PAP group; the participants who exhibited poor cooperation were placed in the supine APP group. Until the number of participants in each group reached 80, the group was terminated. The inclusion criteria were the need for one-time complete chest DR and no aberrant chest radiographs. The exclusion criteria were as follows: inability to cooperate or complete one-time chest DR after enrollment, thoracic radiographs displaying abnormities in the thoracic cage, organic lesions in the heart, space-occupying lesions in the lungs, and abnormal mediastinal shadows in the cardiac silhouette. A total of 248 participants were excluded, and 240 participants were finally included (Fig 1), including 137 males and 103 females. Their ages ranged from 36 to 47 months, with a mean of 41.5±3.5 months. Their heights ranged from 91 cm to 109 cm, with a mean of 99.83±3.55 cm. Their weights ranged from 10.50 kg to 21.00 kg, with a mean of 15.31±1.92 kg. Their BMIs ranged from 11.57 kg/m^2^ to 19.58 kg/m^2^, with a mean of 15.34±1.51 kg/m^2^.

**Fig 1:** Study design flow chart. The numbers in parentheses in the boxes in the first two columns indicate the number of children who underwent chest X-ray radiography. The numbers in the boxes in the remaining eight columns indicate the number of children who were excluded or included. N/A indicates “not applicable”.

### Equipment and methods

This study was performed using two DR imaging systems (Discovery XR656 and Discovery XR650; GE Medical Systems, Milwaukee, WI, USA). Discovery XR656 was installed in the Radiology Department in 2015 and is referred to as unit A, and Discovery XR650 was installed in 2012 and is referred to as unit B. Two 40.64-cm×40.64-cm cesium iodide/amorphous silicon flat-panel detectors were used for the standing and supine projections in the two units [15]. The acquisition matrix was 2022×2022, the pixel size was 200 μm, and the limiting spatial resolution was 2.5 line pairs per millimeter. A diagnostic medical display system (MDNG-3421; Barco, Suzhou, China) was used to evaluate image quality. The following conditions were used for all three groups in the two units: tube voltage, 80 kilovolts (KVs); source-to-image receptor distance (SID), 100 cm; and small focal spot size, 0.6 mm. The inherent filtration provided by the tube housing, collimator, dose-area measuring chamber, and light localizer was equivalent to 3.1 mm of aluminum (Al). Automatic exposure control (AEC) was used for image acquisition when the participant’s abdomen maximally bulged. The irradiation field was minimized as much as possible and included the apexes of the lungs, clavicles, and the costophrenic angle and the edges of the thoracic walls. During DR, the pediatric participant lifted his/her arms with his/her mandible slightly lifted [4] while his/her back or chest was close to the flat-panel detector. The DAP and ESD values provided by the DR units were recorded after every exposure and were used as an indirect evaluation index of the radiation dose [16,17]. The nonirradiated sites of the pediatric participants and their accompanying caregivers were protected [18]. To explore whether some factors influencing the radiation dose exceeded suitable limitations and ensure equipment performance consistency and the reliability and reproducibility of exposure parameters, quality control tests were performed at regular intervals throughout this study by the Medical Physics Department of the hospital [14].

### Image analysis

The chest DR image quality evaluation of pediatric participants was performed by consensus using the VGAS by two experienced pediatric radiologists with 20 and 21 years of experience, respectively, who were blinded to the participants’ clinical information. The image clarity of the trachea and proximal bronchi, the pulmonary blood vessels, the heart and aortic margins, the mediastinum, the vertebrae behind the cardiac silhouette, the diaphragm, and the costophrenic angle was scored using five grades [9]: 1 point, definitely unclear; 2 points, some definitely unclear areas; 3 points, clarity cannot be determined; 4 points, some definitely clear areas; and 5 points, definitely clear. The VGAS for each pediatric participant was the sum of the six aforementioned items (maximum score of 30). The mean VGAS for the 80 participants in each group (40 participants who were imaged using unit A and 40 participants who were imaged using unit B) was taken as the score for that group. A closed curve was plotted along the lung field and the mediastinal margin, and the lung field area (LFA) was then measured. The longitudinal distance (LD) was the distance from the apex of the right lung to the apex of the right diaphragm (Fig 2).

**Fig 2:** Schematic diagram showing LD and LFA measurements in a chest DR image of a pediatric participant. The subject is a 45-month-old female. In the figure, **a** represents the LD from the apex of the right lung to the apex of the right diaphragm, **b** represents the right LFA obtained by measuring the area within the closed curve drawn along the right lung field and the mediastinal margin, and **c** represents the left LFA obtained by measuring the area within the closed curve drawn along the left lung field and the mediastinal margin. The sum of **b** and **c** represents the entire LFA of the participant.

### Statistical analysis

Statistical analyses were performed using Statistical Product and Service Solutions version 24 (IBM Corporation, Armonk, NY, USA). First, the conformation of numeric data to a normal distribution and homogeneity of variance were determined using the Kolmogorov-Smirnov test and Levene’s test, respectively. *P*<0.05 was considered statistically significant for numeric data. Second, differences in age, height, weight, BMI, DAP, ESD, LD, LFA, and VGAS among the supine APP, standing APP, and standing PAP groups were compared using one-way analysis of variance. After *P*<0.05 was obtained using one-way analysis of variance, the least significant difference-*t* test was further used to compare the differences in the abovementioned variables between the three groups in pairs. Third, the chi-square test was used to analyze possible differences related to sex between the supine APP, standing APP, and standing PAP groups. To compare differences in age, BMI, DAP, ESD, LD, LFA, and VGAS between the male and female participants or between unit A and unit B participants, the independent sample *t* test was applied. In addition, the correlations among ESD, DAP, VGAS, and BMI in the three groups were analyzed using the Pearson test. The correlations among ESD, DAP, VGAS, BMI, and sex in the three groups were compared using the Spearman test. *P*<0.05 was considered statistically significant.

## Results

### Comparison of the general status of the pediatric participants in the three groups

Statistically significant differences in DAP, ESD, LD, and LFA were found among the three groups (*P*<0.05). The DAP and ESD values for the standing PAP (Fig 3) and standing APP (Fig 4) groups were significantly lower than those for the supine APP group (Fig 5) (*P*<0.05, respectively), but the LDs for the standing PAP and standing APP groups were significantly higher than that for the supine APP group (*P*<0.05, respectively). No statistically significant differences in DAP, ESD, or LD were found between the standing PAP group and the standing APP group (*P*>0.05). LFA and age were significantly higher in the standing PAP group than in the standing and supine APP groups (*P*<0.05, respectively), but no statistically significant differences in LFA or age were found between the standing and supine APP groups (*P*>0.05, respectively). In addition, no statistically significant differences in sex distribution, height, weight, BMI, or VGAS were observed among the three groups (*P*>0.05) (Table 1).

**Fig 3:** Chest DR image of a pediatric participant in the standing PAP group (unit A). The image shown is that of a 43-month-old male with a height of 104 cm, a weight of 15 kg, and a BMI of 13.87 kg/m^2^. The ESD value was 0.05 mGy, the DAP value was 0.13 dGy•cm^2^, the VGAS was 30, the right LFA was 76.57 cm^2^, the left LFA was 65.20 cm^2^, the total LFA was 141.77 cm^2^, and the LD was 12.36 cm.

**Fig 4:** Chest DR image of a pediatric participant in the standing APP group (unit A). The image shown is that of a 40-month-old female with a height of 105 cm, a weight of 17 kg, and a BMI of 15.42 kg/m^2^. The ESD value was 0.06 mGy, the DAP value was 0.20 dGy•cm^2^, the VGAS was 29, the right LFA was 68.95 cm^2^, the left LFA was 49.82 cm^2^, the total LFA was 118.77 cm^2^, and the LD was 12.77 cm.

**Fig 5:** Chest DR image of a pediatric participant in the supine APP group (unit A). The image shown is that of a 38-month-old female with a height of 109 cm, a weight of 15 kg, and a BMI of 12.63 kg/m^2^. The ESD value was 0.07 mGy, the DAP value was 0.22 dGy•cm^2^, the VGAS was 29, the right LFA was 64.80 cm^2^, the left LFA was 50.50 cm^2^, the total LFA was 115.30 cm^2^, and the LD was 11.50 cm.

**Table 1:** Demographic data, radiation dose, and image quality for the supine APP, standing APP, and standing PAP groups (n = 240).

	n	Sex (m/f)	ESD (mGy)	DAP (dGy•cm^2^)	LFA (cm^2^)	LD (cm)	VGAS	Age (months)	Height (cm)	Weight (kg)	BMI (kg/m^2^)
Supine APP	80	45/35	0.16±0.09	0.55±0.32	101.72±18.56	11.10±1.03	29.21±0.90	41.2±3.5	100.41±3.62	15.27±2.05	15.10±1.43
Standing APP	80	49/31	0.12±0.07^□^	0.42±0.25^□^	106.00±14.34^▲^	11.90±1.09^□^	29.18±1.02	40.9±3.5^▲^	99.25±3.63	15.24±1.94	15.46±1.63
Standing PAP	80	43/37	0.12±0.07^□^^■^	0.41±0.25^□^^■^	120.16±19.76^□^^Δ^	11.95±1.35^□^^■^	29.38±1.00	42.3±3.3^□^^Δ^	99.84±3.34	15.43±1.79	15.46±1.46
*F* or *χ*^*2*^ value		0.95	7.88	6.01	23.77	13.46	0.96	3.83	2.17	0.23	1.56
*P* value		0.62	<0.001	0.003	<0.001	<0.001	0.39	0.02	0.12	0.80	0.21

Note:

^□^ indicates a statistically significant difference compared with the supine APP group (*P*<0.05);

^Δ^ indicates a statistically significant difference compared with the standing APP group (*P*<0.05);

^▲^ indicates no statistically significant difference compared with the supine APP group (*P*>0.05); and

^■^ indicates no statistically significant difference compared with the standing APP group (*P*>0.05).

### Comparison of the general status, radiation dose, and image quality between male and female participants in the three groups

No statistically significant differences in DAP, ESD, VGAS, LFA, BMI, LD, or age were identified between the male and female participants in the three groups (*P*>0.05) (Table 2).

**Table 2:** Demographic data, radiation dose, and image quality for the male and female participants in the three groups (n = 240).

	n	ESD (mGy)	DAP (dGy•cm^2^)	LFA (cm^2^)	LD (cm)	VGAS	Age (months)	BMI (kg/m^2^)
Male	137	0.14±0.08	0.48±0.29	110.62±19.70	11.77±1.20	29.30±0.93	41.3±3.5	15.40±1.55
Female	103	0.13±0.08	0.44±0.26	107.52±18.76	11.50±1.24	29.19±1.02	41.8±3.4	15.26±1.46
*T* value		0.97	1.03	1.23	1.70	0.83	-1.13	0.72
*P* value		0.34	0.31	0.22	0.09	0.41	0.26	0.47

### Comparison of general status, radiation dose, and image quality analysis for participants imaged using unit A with those for participants imaged using unit B

Statistically significant differences in DAP, ESD, and VGAS were found between participants imaged using unit A and those imaged using unit B (*P*<0.05). DAP, ESD, and VGAS for participants imaged using unit A were significantly lower than those for participants imaged using unit B. However, no statistically significant differences in LFA, sex distribution, BMI, LD, or age were observed between the participants imaged using the two units (*P*≥0.05) (Table 3).

**Table 3:** Comparison of the demographic data, radiation dose, and image quality for participants imaged using unit A and unit B (n = 240).

	n	Sex (m/f)	ESD (mGy)	DAP (dGy•cm^2^)	LFA (cm^2^)	LD (cm)	VGAS	Age (months)	BMI (kg/m^2^)
Unit A	120	67/53	0.06±0.01	0.21±0.05	109.95±17.09	11.49±1.10	28.89±0.92	41.1±3.4	15.18±1.35
Unit B	120	70/50	0.20±0.05	0.71±0.17	108.64±21.37	11.81±1.32	29.62±0.88	41.9±3.5	15.50±1.65
*T* or *χ*^*2*^ value		0.15	-32.18	-31.28	0.53	-2.02	-6.22	-1.94	-1.60
*P* value		0.70	<0.001	<0.001	0.60	0.05	<0.001	0.05	0.11

### Analysis of the correlation between ESD, DAP, VGAS, BMI, and sex in the three groups

A statistically significant positive correlation among ESD, DAP, and VGAS was found; larger ESD and DAP values corresponded to higher VGAS values (*P*<0.05, respectively). Additionally, a statistically significant positive correlation among ESD, DAP, and BMI was identified, indicating that higher BMI is associated with larger ESD and DAP values (*P*<0.05, respectively). However, no statistically significant correlation was found between BMI and VGAS (*P*>0.05) or among ESD, DAP, VGAS, BMI, and sex (*P*>0.05) (Table 4).

**Table 4:** Analysis of the correlations between ESD, DAP, VGAS, BMI, and sex in the three groups (n = 240).

	ESD	DAP	VGAS	BMI	Sex
ESD	N/A	R = 0.99 (P<0.001)	R = 0.32 (P<0.001)	R = 0.14 (P = 0.03)	R = -0.06 (P = 0.37)
DAP	R = 0.99 (P<0.001)	N/A	R = 0.31 (P<0.001)	R = 0.16 (P = 0.01)	R = -0.06 (P = 0.36)
VGAS	R = 0.32 (P<0.001)	R = 0.31 (P<0.001)	N/A	R = -0.03 (P = 0.67)	R = -0.05 (P = 0.43)
BMI	R = 0.14 (P = 0.03)	R = 0.16 (P = 0.01)	R = -0.03 (P = 0.67)	N/A	R = -0.04 (P = 0.51)
Sex	R = -0.06 (P = 0.37)	R = -0.06 (P = 0.36)	R = -0.05 (P = 0.43)	R = -0.04 (P = 0.51)	N/A

Note: N/A indicates “not applicable”.

## Discussion

In this study, the DAP and ESD values for the standing PAP and standing APP groups were considerably lower than those for the supine APP group, potentially because under conditions in which the exposure parameters were the same, the heart shadow, the structure of the hilus pulmonis, the diaphragm, and the subdiaphragmatic organs were in a naturally sagging position due to the influence of gravity, thereby decreasing overlaps among the images derived from these structures. Therefore, in a standing projection in children, the current (mAs) required for AEC image collection, which changes and depends on beam attenuation in light of the body habitus of the patient [16], is lower than that required in a supine projection. Although no statistically significant differences in DAP or ESD were found between the standing PAP and APP groups, the radiation dose to superficial organs, such as the breast tissue, may be lower with standing PAP than with standing APP when chest DR is performed [6,19]. In addition, children around the age of three years primarily employ abdominal breathing, during which maximal inhalation occurs when the abdomen is bulging. Thus, in this study, regardless of whether or not the children cooperated during the procedure, exposure was conducted when their abdomens were maximally raised. Generally, as children age, their degree of cooperation also gradually increases. The mean age of the participants in the standing PAP group was significantly higher than that of the participants in the standing and supine APP groups, and this may have led to better cooperation among the participants in the standing PAP group than in the standing and supine APP groups and a higher degree of inspiration in the PAP group. This finding is consistent with the higher LD and the significantly larger LFA observed for the PAP group in comparison with the APP groups. In addition, no statistically significant differences in VGAS were found among the three groups, showing that the image quality of all three projections meets diagnostic requirements. These results suggest that the use of standing PAP can decrease the radiation dose and fully display the lung field in 3- and 4-year-old children.

No statistically significant differences in DAP or ESD were noted between the male and female participants in this study; this finding is not consistent with previous research results indicating that the radiation dose received by adult males was significantly higher than that received by adult females [14]. This finding may result from the lack of difference in BMI between the male and female pediatric participants in this research, in which exposure conditions were consistent, and the small sample size; thus, further validation of this result is needed. Moreover, the DAP and ESD values obtained using unit A were significantly lower than those obtained using unit B. Because the flat-panel detectors and exposure conditions were the same in the two imaging units and there were no differences in sex distribution, BMI, or age between the participants who were imaged using the two units, the observed difference in radiation dose may be related to the service lives of the units. Unit B has been in use longer than unit A (the two systems were installed in 2012 and 2015, respectively). However, the VGAS obtained using unit A was significantly lower than that obtained using unit B; this is consistent with the positive correlation between VGAS, ESD, and DAP and suggests that a higher radiation dose corresponds to better image quality.

Furthermore, no statistically significant differences in sex distribution, height, weight, or BMI were found among the supine APP, standing APP, and standing PAP groups, indicating that the analysis of radiation doses for chest DR in 3- and 4-year-old children is valid when previously validated exposure parameters are applied. Some researchers have suggested that in children, the DAP values obtained on chest DR decrease as SID decreases; however, a shorter SID results in a higher ESD value [6]. Other academicians have found that the combined application of 0.6-mm focal spots and SID greater than 100 cm can objectively reflect heart size and control penumbra blurriness, hence guaranteeing image clarity [4,5,16,18]. Therefore, a SID of 100 cm was adopted in this study. Moreover, a previous study indicated that in rabbits, the application of 2-mm Al inherent filtration (simulating the neonatal chest) in computed radiography units may decrease the ESD value by 53.4% while not affecting image quality [8]. Considering that the chest thickness of 3- and 4-year-old children is greater than that of rabbits and that insufficient X-ray beam filtration may result in greater participant exposure [14,20], inherent filtration of 3.1-mm Al was applied in our study to further reduce the ESD value during chest DR. In our study, the DAP values for the standing PAP, supine APP and standing APP groups were higher than the value of 0.22±0.07 dGy•cm^2^ obtained for a group of 3- to 7-year-old children in a previous study [7], although 80 kV and AEC were also used in the latter group. Furthermore, some academicians have found that the optimizing exposure parameters for chest DR in 1- to 5-year-old children (using equivalent phantoms) are 81 kV and 2.0 mAs, and the ESD value is 0.08 mGy [21]. In our study, the ESD values for the standing PAP, supine and standing APP groups were higher than those reported in the aforementioned research. These results indicate that 80 kV and AEC are the optimal exposure conditions for chest DR in 3- and 4-year-old children; this result should be further validated in the future. In addition, the use of AEC can avoid subjective differences by operators and control the exposure dose [15,22,23].

This study has some limitations. First, we selected only 3- and 4-year-old children, and the sample size was small. Comparisons between different KVs and SIDs were not made. In future studies, the age range and sample size will be expanded, and different KVs and SIDs will be compared. Second, in this study, we employed only GE Discovery XR656 and XR650 cesium iodide/amorphous silicon flat-panel detectors, but differences in materials, structure, and processes between flat-panel detectors from different manufacturers or different types of flat-panel detectors may result in differences in detective quantum efficiency [24] and spatial resolution, thereby resulting in differences in exposure parameters. In future studies, we will compare the differences in image quality and radiation dose that may result from the use of flat-panel detectors of different types and from different manufacturers. Third, to exclude any possible bias, only children without abnormal chest radiographs were included in this study. In the future, we will further explore the effects of different photography projections on chest DR in children with various diseases.

## Conclusions

When choosing an imaging projection for chest DR for 3- and 4-year-old children, diagnostic requirements should not be the only consideration; the individual’s status should also be considered. Standing PAP should be the preferred projection choice, followed by standing APP and supine APP, because standing PAP can decrease the radiation dose received during chest DR.

## Supporting information

S1 Table Raw data for each participant in the three groups (n = 240). This table provides the raw demographic data, radiation dose, and image quality for each participant in the supine APP, standing APP, and standing PAP groups.
(XLSX)
